The article "Study on the Current Status and Influencing Factors of Workplace Violence to Medical Staff in Intensive Care Units" was retracted in 2023. Reasons: signs of a paper mill; suspected computer-generated content; unreliable results or conclusions; lack of ethics approval or compliance.

# Study on the Current Status and Influencing Factors of Workplace Violence to Medical Staff in Intensive Care Units

**DOI:** 10.1155/2022/1792035

**Published:** 2022-06-17

**Authors:** Xingke Yi, Xiuchan Feng

**Affiliations:** The Second Affiliated Hospital, Department of Critical Care Medicine, Hengyang Medical School, University of South China, Hengyang, Hunan 421001, China

## Abstract

**Objective:**

To explore the current status and influencing factors of workplace violence to medical staff in intensive care unit (ICU).

**Methods:**

A total of 230 medical staff in the ICU of Hengyang city were enrolled as the research subjects between October 2021 and January 2022. The situations and characteristics of workplace violence were collected with questionnaires. The influencing factors of workplace violence were analyzed by univariate and multivariate logistic regression analyses.

**Results:**

The incidence of workplace violence to ICU medical staff was 40.43%. There were 18.70% of them threatened, 13.48% with verbal violence, 10.00% with physical violence, and 7.39% with sexual harassment. Of the 114 workplace violence incidents, there were 69 (59.65%) during the day, 101 (88.60%) only with medical staff on the spot, and 91 (79.82%) with male perpetrators (mainly on patients and their families). The main reasons for violence were verbal miscommunication (15.79%), too long waiting time for treatment (27.19%), and unsatisfactory treatment effect (38.60%). The main coping style of medical staff after suffering violence was patient explanation (64.04%). Multivariate regression analysis showed that working years ≤5 years (OR = 2.093, *P*=0.009) and weekly working time >45 h (OR = 2.127, *P*=0.022) were independent risk factors of workplace violence to ICU medical staff.

**Conclusion:**

The working years ≤5 years and weekly working time >45 h are high-risk factors of workplace violence to ICU medical staff. The hospital can prevent and control workplace violence based on the high-risk factors to reduce the incidence of workplace violence.

## 1. Introduction

Workplace violence refers to abuse, threats, humiliation, or attacks in the workplace, including verbal and physical violence. Research indicates that workplace violence is one of the major health risk factors for people working in the workplace and that such behaviors can lead to a variety of psychological and emotional conditions that affect job quality [1, 2]. Hospitals are places where workplace violence occurs frequently. According to relevant statistics, more than 50% of emergency nurses in the world have experienced workplace violence and most of the violence comes from patients [3, 4]. However, most medical staff adopt negative coping styles to deal with workplace violence, which has caused some harm to their professional attitude and mental health [5]. Studies by Yuan et al. pointed out that workplace violence has a serious adverse effect on the mental health of the medical staff, causing nurses to produce psychological stress reactions such as anger, depression, and anxiety [6]. In addition, the frequent occurrence of psychological violence can also produce qualitative changes, resulting in the decline of the overall job satisfaction rate of medical staff, resulting in the deterioration of hospital medical quality. Survey data showed that young nurses under 35 were more likely to experience workplace violence when working alone due to lack of experience [7, 8]. Most of the current research focuses on the emergency department, psychiatry, and other groups, and there are few research studies specifically on the workplace violence of intensive care unit (ICU) medical staff. The ICU is a high-risk area for workplace violence in hospitals because patients are critically ill, have a high mortality rate, and are prone to delirium; most of their family members have anxiety, irritability, and other negative emotions, and the probability of workplace violence is also greatly increased [9]. This study analyzes the current situation and characteristics of workplace violence suffered by medical staff in intensive care units in order to provide a basis for guiding targeted prevention and control measures.

## 2. Materials and Methods

### 2.1. General Information

From October 2021 to January 2022, 230 medical staff in the ICU of Hengyang city were selected as the research subjects. All the enrolled personnel were 27 males and 203 females; their ages ranged from 22 to 45 years, with an average of (28.76 ± 4.83) years. In terms of education background, 36 research subjects graduated from junior colleges, 161 were undergraduates, 27 had a master's degree, and 6 were doctors. 122 subjects have primary titles, 82 subjects have intermediate titles, and 26 subjects have senior titles; 100 subjects have worked for more than 5 years, and 130 subjects have worked for ≤5 years; 114 subjects were unmarried, and 116 were married; 31 cases were the only child in their families, while 199 subjects were opposite; 171 cases had weekly working hours >45 h, and 59 cases had ≤45 h. This study complies with the requirements of the World Medical Association Declaration of Helsinki.

### 2.2. Inclusion Criteria

The inclusion criteria were as follows: ① regular employees working in the intensive care unit of our hospital; ② ICU medical staff who have access to patients; ③ those who gave informed consent and voluntary participation in the survey.

### 2.3. Exclusion Criteria

The exclusion criteria were as follows: ① interns in the ICU; ② those who are leaving the job for more than 3 months due to maternity leave and other reasons; ③ medical staff in the neonatal ICU; ④ those who have provided incomplete questionnaire data; ⑤ those who have worked in the ICU for less than 1 year.

### 2.4. Methods

All participants were surveyed using a questionnaire on workplace violence made by our hospital. The questionnaire included age, gender, education background, job title, length of service, marital status, if they were the only child in their families, and weekly working hours. The characteristics of workplace violence suffered by ICU medical staff were counted and recorded, including the time of occurrence, time being alone, gender of the perpetrator, age of the perpetrator, identity of the perpetrator, reasons for the violence, and ways of coping with the violence.

### 2.5. Observation Indicators

The observation indicators included the following: (1) statistical analysis of workplace violence suffered by ICU medical staff; (2) statistical analysis of the characteristics of workplace violence incidents suffered by ICU medical staff; (3) univariate analysis of the influencing factors of workplace violence among ICU medical staff; (4) multivariate analysis of independent influencing factors of workplace violence incidents suffered by ICU medical staff.

### 2.6. Statistical Processing

SPSS 18.0 was used to process data, count data were expressed as percentage (%), *χ*^*2*^ test was conducted, and univariate and multivariate logistic regressions were used to analyze the influencing factors of workplace violence suffered by ICU medical staff. *P* < 0.05 shows that the difference is statistically significant.

## 3. Results

### 3.1. Workplace Violence Suffered by ICU Medical Staff

Among the 230 ICU medical staff, 93 (40.43%) staff suffered workplace violence, 18.70% staff suffered threats, 13.48% staff suffered verbal violence, 10.00% staff suffered physical violence, and 7.39% staff suffered sexual harassment. A total of 114 workplace violence incidents occurred, as shown in Table 1.

### 3.2. Characteristics of Workplace Violence Incidents Suffered by ICU Medical Staff

Among the 114 workplace violence incidents, 69 (59.65%) occurred during the day, 101 (88.60%) medical staff were present alone, and 91 (79.82%) perpetrators were male, and the perpetrators were mainly patients and their families. The main reasons for the violence were wrong verbal communication (15.79%), long time waiting for treatment (27.19%), and unsatisfactory treatment effect (38.60%). The main coping method of the medical staff after violence was patient explanation (64.04%), as shown in Table 2.

### 3.3. Univariate Analysis of the Influencing Factors of Workplace Violence That ICU Medical Staff Suffered

According to the workplace violence suffered by the ICU medical staff, they were divided into a violence group and a nonviolence group. There was a statistically significant difference between the two groups of medical staff in terms of working years and weekly working hours (*P* < 0.05). There was no statistically significant difference in gender, age, education background, job title, and marital status and if they were the only child in their families (*P* > 0.05), as shown in Table 3.

### 3.4. Multivariate Analysis of the Influencing Factors of Workplace Violence That ICU Medical Staff Suffered

Assigning scores to the variables with statistical significance in Table 3, violence group = 1, nonviolence group = 0; length of service > 5 years = 0, length of service ≤ 5 years = 1, weekly working hours >45 h = 1, and weekly working hours ≤ 45 h = 0 and using multivariate logistic analysis, working age ≤5 years (OR = 2.093, *P*=0.009) and weekly working time >45 h (OR = 2.127, *P*=0.022) were independent risk factors for ICU medical staff suffering workplace violence, as shown in Table 4.

## 4. Discussion

Hospital workplace violence has become an important health problem that endangers the physical and mental health of medical staff worldwide [10]. According to the report of Indian Medical Association, 75% of doctors have experienced violence, while ICU accounts for nearly half of the total, and ICU medical staff face such incidents almost every day [11]. Therefore, how to optimize the diagnosis and treatment process, close the doctor-patient relationship, and then prevent the violence in the hospital workplace have become the key and difficult problem facing the hospital construction.

In this study, 40.43% of ICU medical staff suffered from workplace violence, which is similar to what Chu Haitao et al have found [12]. Among them, 18.70% had experienced threats, 13.48% had experienced verbal violence, 10.00% had experienced physical violence, and 7.39% had experienced sexual harassment, indicating that threats and verbal violence were the main types of workplace violence in the ICU. Patients and their family members used these irrational ways to protect their rights, which showed that the hospital's relevant management and national rights protection laws and regulations were weak. When medical staff are busy or exhausted and fail to meet the requirements of patients and their family members in time, patients and their families are prone to emotional agitation, which in turn leads to violent incidents. Therefore, violence in the ICU workplace mainly occurred during the daytime, which is the peak period for family visits of patients and the main time for medical staff to check the condition of patients. Previous research have shown that refusing the unreasonable demands of patients or their family members is the main reason why medical staff are subjected to violence in hospital workplaces, which is related to the imbalance between the supply and demand of medical services in the country [13]. 88.60% of the workplace violence occurred when medical staff were alone, prompting medical staff to be more vigilant and try to avoid ICU workplace violence caused by vulnerable situations such as being alone. Most of the perpetrators were middle-aged men. Because the men at this stage bear the dual pressures of work and life, they may be in adverse states such as anxiety and irritability for a long time and have poor tolerance for complicated medical procedures, long-time queuing examination, unsatisfactory treatment effect, etc. Therefore, such patients and their family members are more likely to be triggered by violence.

Wang et al. found that positive coping and negative coping had a great impact on the psychological stress level of Chinese medical staff and played a mediating role in stress perception and psychological distress [14]. Through a survey of Chinese nurses, Ding et al. found that negative coping played a mediating role between self-efficacy and emotional exhaustion and had a negative effect on the degree of emotional exhaustion of Chinese medical staff [15]. In this study, the main coping method of medical staff after being subjected to violence was patient explanation. The main reason is that this method can help hospitals establish a safe and orderly working environment. But the downside is that it will put enormous pressure on medical staff. Under the influence of the violence of patients and their family members, the ICU medical staff are prone to anxiety, depression, and other negative psychology and may even develop posttraumatic stress disorder without timely intervention. However, only 9.65% of medical staff chose to report to the police/public prosecution, indicating that the hospital's alarm channel was not smooth and the hospital needed to strengthen the violence prevention equipment, such as monitors and alarms, and should also add relevant departments to solve violent incidents to facilitate medical staff to seek help and resolve contradictions.

Medical staff with short working experience are inexperienced, they have less participation in hospital-related safety training, and they have insufficient understanding of the regulations for preventing workplace violence. In addition, frequent medical troubles and tense doctor-patient relationship in recent years have led to a significant increase in the risk of hospital violence among medical staff. In this case, the medical staff do not have enough time to form a good doctor-patient relationship with patients, and communication between the two parties is difficult, which increases the probability of workplace violence in the ICU. The study by Liu Yuan et al. found that job burnout was one of the factors that caused the tension between doctors and patients [16]. So our study showed that working age ≤5 years and weekly working hours >45 h were independent risk factors for ICU medical staff in experiencing workplace violence. In addition, the medical staff have been in a tense environment between doctors and patients for a long time, and they are more vigilant for medical patients, which greatly reduces the contact and communication between doctors and patients and further increases the risk of hospital violence [17].

To sum up, length of service ≤5 years and weekly working hours >45 hours are high-risk factors for the workplace violence suffered by ICU medical staff. Hospitals can prevent and control these high-risk factors to reduce the incidence of workplace violence in the ICU. However, the sample size of this study was not large, and some of the observed insignificant associations (such as education and age) may be caused by insufficient samples. In addition, the subjects of this study were recruited by sampling, which may lead to bias in individual factors, and the true rate of some factors (such as working hours per week) may be underestimated.

## Figures and Tables

**Table 1:** Workplace violence suffered by ICU medical staff.

Type of violence	Number of staff	Composition ratio (%)
Threat	43	18.70
Verbal violence	31	13.48
Physical violence	23	10.00
Sexual harassment	17	7.39
Total	93	40.43

**Table 2:** Characteristics of workplace violence incidents suffered by ICU medical staff.

Characteristics of workplace violence incidents		Case	Composition ratio (%)
Time of occurrence	Day shift	68	59.65
	Night shift	39	34.21
	After work	7	6.14

If they were present alone	Yes	101	88.60
	No	13	11.40

Gender of perpetrators	Male	91	79.82
	Female	23	20.18

Age of perpetrators	<18 years old	1	0.88
	18∼40 years old	13	11.40
	41∼60 years old	74	64.91
	>60 years old	26	22.81
	Patients	60	52.63

Identity of perpetrators	Family members of patients	49	42.98
	Other people	5	4.39
	High treatment costs	9	7.89
	Death of patients	12	10.53

Reason for workplace violence	Wrong verbal communication	18	15.79
	Long waiting time for treatment	31	27.19
	Unsatisfactory treatment effect	44	38.60
	Patient explanation	73	64.04

Coping method	Language warning	28	24.56
	Terminating treatment	2	1.75
	Calling the police/prosecuting	11	9.65

**Table 3:** Univariate analysis of the influencing factors of workplace violence that ICU medical staff suffered.

Item	*n*	Violence group (*n* = 93)		Nonviolence group (*n* = 104)		*χ* ^*2*^	*P*
		Case	Proportion	Case	Proportion		
Gender						1.483	0.223
Male	27	8	8.60	19	13.87		
Female	203	85	91.40	118	86.13		

Age (year)						1.309	0.253
>30	60	28	30.11	32	23.36		
≤30	170	65	69.89	105	76.64		

Education background						0.070	0.792
Junior college and undergraduate	161	66	70.97	95	69.34		
Master's degree and above	69	27	29.03	42	30.66		

Job title						0.976	0.323
Primary	122	53	56.99	69	50.36		
Intermediate and senior	108	40	43.01	68	49.64		

Length of service						6.539	0.011
>5	100	31	33.33	69	50.36		
≤5	130	62	66.67	68	49.64		

Marital status						0.262	0.609
Unmarried	114	48	51.61	66	48.18		
Married	116	45	48.39	71	51.82		

If they were the only child in their families						0.941	0.332
Yes	31	15	16.13	16	11.68		
No	199	78	83.87	121	88.32		

Weekly working hours (h)						5.842	0.016
>45	171	77	82.80	94	68.61		
≤45	59	16	17.20	43	31.39		

**Table 4:** Multivariate analysis of the influencing factors of workplace violence that ICU medical staff suffered.

Indicator	*β*	SE	Wald *χ*^*2*^	OR	95% CI	*P*
Length of service (≤5 years vs >5 years)	0.738	0.282	6.839	2.093	1.203∼3.639	0.009
Weekly working hours (>45 h vs ≤45 h)	0.755	0.331	5.214	2.127	1.113∼4.066	0.022

## Data Availability

The data can be obtained from the corresponding author upon reasonable request.

## References

[1] Giménez Lozano J. M., Martínez Ramón J. P., Morales Rodríguez F. M. (2021). Doctors and nurses: a systematic review of the risk and protective factors in workplace violence and burnout. *International Journal of Environmental Research and Public Health*.

[2] Pol A., Carter M., Bouchoucha S. (2019). Violence and aggression in the intensive care unit: what is the impact of Australian national emergency access target?. *Australian Critical Care*.

[3] Wang J. J., Lv H., Xing X. L. (2021). A cross-sectional study on the incidence and risk factors of workplace violence among medical workers in China. *Medicine in Society*.

[4] Gai J. X., Gao H., Ren X. Y. (2021). Visual analysis of research on workplace violence in emergency nursing based on citeSpace. *Chinese Journal of Modern Nursing*.

[5] Chen N., Zhang M., Li R. (2021). Investigation of workplace violence response measures in a second-class hospital. *China Occupational Medicine*.

[6] Yuan Y., Sun W. (2021). The impact of workplace violence on post-traumatic stress in emergency department nurses. *Occupation and Health*.

[7] Li R., Yang J., Lv Y. L. (2020). Investigation on the correlation between empathy fatigue and hospital workplace violence among medical staff. *Journal of Xinxiang Medical College*.

[8] Huang Y. M., Zhang M., Li R. (2021). Analysis on the current situation and influencing factors of psychological violence suffered by medical workers in a second-class hospital. *Chinese Journal of Occupational Medicine*.

[9] Munta K., Harde Y., Kumar N. S., Kumar J. R., Rao S. M., Dnyaneshwar M. (2019). A survey on workplace violence experienced by critical care physicians. *Indian Journal of Critical Care Medicine*.

[10] Zhou T. T., Huang P., Chen Q. J. (2020). Status and influencing factors of workplace violence suffered by emergency nurses in tertiary hospitals in Jiangsu Province. *Chinese Journal of Modern Nursing*.

[11] Joshi S. C., Joshi R. (2018). Doctor becomes a patient: a qualitative study of health care work place violence related perception among junior doctors working in a teaching hospital in India. *International Journal of Community Medicine and Public Health*.

[12] Chu H. T., Wei X. J., Li L. M. (2021). Analysis of workplace violence among nurses in the intensive care unit of a tertiary general hospital in Henan Province. *Environmental and Occupational Medicine*.

[13] Zhao J. H., Hu L. L., Qin B. (2021). Institutional survey results of improving medical service evaluation in tertiary public hospitals in my country: 2018-2020. *Chinese Journal of Hospital Management*.

[14] Wang Y., Wang P. (2019). Perceived stress and psychological distress among Chinese physicians. *Medicine*.

[15] Ding Y., Yang Y., Yang X. (2015). The mediating role of coping style in the relationship between psychological capital and burnout among Chinese nurses. *PLoS One*.

[16] Liu Y., Liu G. X. (2020). Research on the status quo and related factors of clinician burnout. *Journal of the Third Military Medical University*.

[17] Wang S. Q., Jiang Q. Q., You Q. Q. (2022). Comparison of the status quo and influencing factors of job satisfaction among general practitioners and specialists in my country. *New Medical Knowledge*.

